The article "Comparative study of instrumental measurement and sensory evaluation methods for the repairing effect of mildly damaged hair bundles" was published in 2023. Journal: Skin Res Technol.

# Comparative study of instrumental measurement and sensory evaluation methods for the repairing effect of mildly damaged hair bundles

**DOI:** 10.1111/srt.13394

**Published:** 2023-07-12

**Authors:** Yanwen Jiang, Zhongmou Xu, Yuchen Qiu, Xiaomin Zheng

**Affiliations:** ^1^ Shanghai China‐Norm Quality Technical Service Co., Ltd. Shanghai China; ^2^ Sethic (Guangzhou) Research & Development Center Co., Ltd. Guangzhou China

**Keywords:** ex vivo test, friction factor of hair cuticle, gloss, hair repairing effect, mildly damaged hair

## Abstract

**Objective:**

This study explores the applicability and scientific accuracy of instrument measurements in repairing hair products on slightly damaged hair bundles.

**Materials and method:**

Sixty hair bundles mildly damaged with hydrogen peroxide and ammonia standards were divided into two groups: the treatment and control groups (30 hair bundles each). The treatment group used commercial hair care essential oil, whereas the control group used tap water to treat the damage. The two groups were measured using an instrument before and after the product application. The objective indicators included the gloss of hair, along with hair cuticle dynamic friction coefficient, and against hair cuticle dynamic friction coefficient. At the same time, two evaluators conducted sensory evaluations on the gloss and frizz levels of the hair bundles. Therefore, data comparison and verification were carried out together with instrumental measurement data.

**Results:**

We verified that the instrumental measurement methods could obtain data trends that are consistent with sensory assessment methods; hence, they have the advantages of accuracy, convenience, and quantifiability.

**Conclusion:**

Thus, the instrumental measurement methods we verified can provide objective evidence for the efficacy of hair care products in repairing hair.

## 1 INTRODUCTION

Hair has always occupied a place in the history of humans who pursue beauty. Due to the influence of European and American cultures and Japanese and Korean trends, diverse hair colors are also popular. Asian hair is mostly brown; hence, to obtain more hair color, the first step is to recede the melanin in the hair. However, the current market uses oxidation to destroy the disulfide bond in hair proteins and change the characteristics of the hair surface to achieve fading. Destruction of the protein structure is followed by a reduction in the performance of hair fibers.^1^ Human hair is composed of approximately 80% alpha keratin, which is closely related to its strength, flexibility, durability, and other properties. In pursuit of colorful and diverse hairstyles, these proteins are also damaged to varying degrees, resulting in dull, dry, and easy‐to‐break hair.^2^ Currently, consumers are paying increasing attention to hair repair and maintenance; thus, the demand for such products is also increasing. From hair conditioners to hair masks, fast and easy‐to‐use hair lotions, and essential oils, many brands continue to launch all kinds of hair care products to meet the needs of consumers. Regardless of the dazzling product ad, the real effect is what consumers care most about.

The article "Comparative study of instrumental measurement and sensory evaluation methods for the repairing effect of mildly damaged hair bundles" was published in 2023. Journal: Skin Res Technol.

We can evaluate the effect of hair repair on both subjective and objective aspects. In principle, self‐assessment questionnaires of consumers and sensory assessments conducted by evaluators are subjective. Objective assessment methods include physical instrumental measurement, biological and chemical analysis, and other methods. The evaluation of a product by consumers is greatly influenced by subjective judgment. Based on the American customer satisfaction model, such as the psychological suggestion generated by some well‐known brands or the trust in a product generated by the recommendation of relatives and friends, will increase the expectations of the customers, resulting in a biased evaluation. Although external psychological factors are excluded from the results of professional sensory evaluators, there may be differences between the evaluators. From a rigor of product effect evaluation perspective, instrument measurements are more accurate than sensory evaluations. In addition, the hair texture of different people is also different. Therefore, it is biased to rely solely on subjective judgment to evaluate a product. If combined with instrument measurements, the efficacy of test results of hair care products can be more objective.

There are many objective methods for the direct qualitative and quantitative detection of chemical hair bundle damage, such as determining metal ion adsorption or protein loss.^3^ However, the instruments and reagents used are usually utilized by scientific research institutions, colleges, and universities and are less likely to be used in efficacy testing. The state of hair cuticle can be presented by friction properties and glossiness data to evaluate the degree of damage to the hair bundle. In a healthy hair state, the cuticle of the hair stem of the hair bundle is arranged neatly and smoothly. When the hair is arranged orderly, and the surface of the hair bundle is relatively flat, the hair appears shiny. On the contrary, when the hair surface becomes rough due to damage to the hair cuticle, light scattering occurs to a large extent, causing the hair to lose its luster.^4^ After the hair bundle was damaged, the surface of the hair cuticle was warped, which significantly affected the dynamic friction factor of the hair bundle. Using the dynamic friction factor, we can objectively calculate the smoothness of hair bundle epidermal hair cuticles. The purpose of measuring the dynamic friction coefficient of hair is not only to quantify damage to the hair surface but also to investigate the attachment and residues of the product on the hair surface.^5^ At the same time, detecting hair bundle friction performance and gloss‐related equipment indicators is more common, easy to obtain, and universal.

The article "Comparative study of instrumental measurement and sensory evaluation methods for the repairing effect of mildly damaged hair bundles" was published in 2023. Journal: Skin Res Technol.

This study aimed to verify the scientific nature of ex vivo quantitative testing methods. The friction performance and glossiness of the hair bundle were measured to objectively evaluate the repair function of hair oil and compared with the corresponding sensory evaluation indexes, glossiness, and smoothness. The scientific nature of the ex vivo quantitative testing methods was confirmed by comparing the trend of instrumental measurement data with clinical evaluation results.

## 2 MATERIALS AND METHODS

### 2.1 Materials and facility

A total of 60 hair bundles were divided into two groups (30 bundles for each group): 30 in the non‐treatment control group and 30 in the test group. Thirty is a common sample size in statistics, known as the moderate sample size. Using 30 samples can provide a relatively robust statistical inference. Similarly, in experiments, a critical factor that affects the model results is the consistency of the hair bundle. Consistency of the hair bundles needs to be considered in various aspects, including the source of the hair, the processing method, the preparation method, and the environmental conditions of the test. By controlling the hair bundles with consistent methods and standards, the errors of test could be minimized, and the reliability and reproducibility of the results should be improved.

The hair bundles used in this study were all human‐isolated hair bundles from the same source and were prepared and cut with same methods to ensure that the shape and size of the test bundles were consistent (natural black Chinese/25 cm × 2.5 cm × 6 g, free 22.5 cm).

For study of hair repair efficacy, slight damage (alkali solubility value is 5%–15%)^6^ to hair bundles was sufficient to demonstrate the efficacy of the product. However, when the hair bundles were more severely damaged, there may be large areas of missing hair cuticles or damage to the hair cortex, which cannot be repaired by the product easily, and may affect the accuracy and reliability of the results. On the contrary, the slightly damaged hair bundles could better control the variables, and the results should be more reproducible and comparable.

The article "Comparative study of instrumental measurement and sensory evaluation methods for the repairing effect of mildly damaged hair bundles" was published in 2023. Journal: Skin Res Technol.

The hair bundles used in this study were treated with hydrogen peroxide and ammonia standards to achieve a slightly damaged state.

Before testing, all hair bundles should be cleaned and pretreated separately using the same method. All hair bundles were soaked in the same shampoo and washed and treated using the same method to ensure that the state of the hair bundles was consistent. After that, all the hair bundles were stored under the same environmental conditions to avoid the impact of changes in environmental conditions.

### 2.2 Hair scales

Hair scales are made up of many tiny scales that cover the surface of the hair and protect its internal structure. When the hair is damaged, the scales may become uneven or even split. The uneven surface of the hair scatters the reflected light, causing hair to appear tarnish and dull, and the rough surfaces also lead to increased friction. The specular reflection and physical friction of the hair can reflect the unevenness of the hair surface and the damage to the hair scales.

### 2.3 Hair gloss by Glossymeter GL200

Glossymeter GL200 (Courage + Khazaka, Köln, Germany) was used to measure the gloss of hair bundles before and after treatment. Three measurements were performed at the top, middle, and end of each bundle. The mean value was obtained after removing the outliers, and the difference in the gloss before and after the treatment was calculated. Glossymeter and SAMBA Hair are common instruments for measuring the gloss of a hair bundle. SAMBA Hair uses a polarization imaging sensor to continuously capture two parallel and cross‐polarization images of the bundle to obtain specular and diffuse images and then calculates the gloss of the bundle by analyzing the intensity and sharpness of the specular and fully reflected light bands in the image. This method is closer to the visual perception evaluation of an evaluator.^7^ The measurement of a glossymeter is based on the reflection of light sent to the skin. Parallel white light was generated by the light‐emitting diodes in the probe head. To emit light at 60° in a relatively small and uniquely designed measurement head, light is sent out at 0° and reflected by a mirror at 60°. Two separate measurement channels were used to measure reflected light. The directly reflected light was again guided by a mirror at 60° into the reflection channel. The scattered/diffuse reflected light was measured at 0°. Diffuse scattering correction can deduct the diffuse light entering the gloss channel through a special formula to obtain a gloss value that is almost unaffected by the hair color.^8^ These results are closer to the physical gloss definition and can more accurately express the improvement in hair cuticles. Therefore, this study used a glossymeter as an instrument to measure the glossiness of hair bundles.

The article "Comparative study of instrumental measurement and sensory evaluation methods for the repairing effect of mildly damaged hair bundles" was published in 2023. Journal: Skin Res Technol.

### 2.4 Hair dynamic friction by MTT175

MTT175 (Dia‐Stron, Hampshire, UK) instrument was used to measure the dynamic friction coefficient before and after hair bundle treatment, and the change between before and after treatment was also calculated. The dynamic friction coefficient is divided into the dynamic friction coefficient along the hair cuticle and the dynamic friction coefficient against the hair cuticle. There are many objective methods for measuring hair properties in the market, and the friction component of MTT175 is a relatively mature method for objectively measuring the friction properties of fibers. When measuring the dynamic friction coefficient of fibers with a directional surface structure, the dynamic friction coefficients of different directions differ. For example, the hair surface has cuticles, and the arrangement of the cuticles is directional. Therefore, when the friction performance of a hair bundle is studied to determine the dynamic friction coefficient, the difference between the long and against hair cuticles should be considered.^9^ The frictional properties of hair cuticles indicate the smoothness of the bundle. The lower friction coefficient/work of the hair cuticles indicates that they are neatly and smoothly aligned. However, based on the frictional properties of the hair cuticles, the lateral hair cuticles are warped after damage to the hair bundle, which leads to an increase in the friction coefficient/work of the hair cuticles. Therefore, in this experiment, the friction performance of the hair bundle was evaluated on both sides of the hair cuticles, along and against them. The instrument measured the dynamic friction coefficient before and after the test product application.

### 2.5 Sensory assessment

The glossiness and smoothness of all bundles were assessed sensorially by two evaluators without any knowledge of the grouping. Two bundles (test and control groups) were compared each time simultaneously, and the evaluator did not inform the condition of grouping. A single light source was used to illuminate the hair bundle directly above. The intensity and width of the highlight band in the isolated hair bundle were used to evaluate the glossiness. The difference between the non‐treatment control and test groups was recorded. To eliminate visual interference, the evaluator wore an eye mask during the smoothness evaluation. The difference in smoothness between the non‐treatment control group and the test group was dictated by the evaluator, and the results were recorded by an assistant. Score 1 was assigned if there was a difference between the test group and the non–treatment control group, and Score 2 was assigned when the difference between them was statistically signficant. When the parameters related to the hair bundle of the test group were better than those of the non‐treatment control group, the difference was positive; otherwise, the difference was negative.

The article "Comparative study of instrumental measurement and sensory evaluation methods for the repairing effect of mildly damaged hair bundles" was published in 2023. Journal: Skin Res Technol.

### 2.6 Implementation

A total of 60 bundles were divided into two groups: 30 in the non‐treatment control group and 30 in the test group.

All bundles were rinsed with water, and a Standard Shampoo (3.0% Sodium Laureth Sulfate (SLES))^10^ was used according to the weight of the dry bundles. After gently rubbing for 30 s (ensure a uniform foam), the bundles were rinsed until there was no foam. The bundles were then soaked in deionized water. After 30 min, the bundles were drained and air‐dried overnight (the bundles were left at a well‐controlled environment temperature [21 ± 1°C] and humidity [50% ± 10%] for 16–24 h). Then, the baseline glossiness and dynamic friction coefficient along and against the hair cuticle were measured for all hair bundles.

### 2.7 Test products

The test product (Förtro Ultimate Repairing Hair Oil, Hua An Tang Group Biotech Co., Ltd., Guangdong, China) was applied evenly to dry hair bundles, and the non‐treatment control group was applied with water. After that, the hair bundles were air‐dried overnight (the bundles were left at a well‐controlled environment temperature [21 ± 1°C] and humidity [50% ± 10%] for 16–24 h). Then, the instrument was used to measure the glossiness and dynamic friction coefficient along hair cuticle and against hair cuticle of all hair bundles.

### 2.8 Descriptive statistics

The descriptive statistics include the number of valid samples (*N*), the mean value (mean), the standard deviation, the standard error, and the improvement rate (vs. baseline) %.

### 2.9 Differential statistics

All data difference tests are conducted using two‐tailed tests, and the significance level is set at *α* = 0.05.

The difference statistics include comparisons of time‐point differences and between‐treatment differences. For time‐point and treatment difference comparisons, analysis of variance (paired *t*‐test) was used.

Comparison between time‐points: before versus after treatment.

Comparison between treatments: test treated versus non‐treatment control.

## 3 RESULT

### 3.1 Results of glossiness

The instrument measured the gloss values before and after the test product application. The larger the difference after‐test product application (T1) and baseline (T0), the better the gloss improvement. The results are illustrated in Table 1 and Figures 1 and 2.

The article "Comparative study of instrumental measurement and sensory evaluation methods for the repairing effect of mildly damaged hair bundles" was published in 2023. Journal: Skin Res Technol.

**TABLE 1:** Gloss—instrumental measurement.

		Time‐point	
	*N*	T0 (baseline)	T1
Mean ± SE			
Test product	30	2.90 ± 0.02	3.38 ± 0.02
Non‐treatment control	30	2.97 ± 0.01	3.02 ± 0.03
Change from baseline (mean ± SE)			
Test product	30		0.48 ± 0.02
Non‐treatment control	30		0.05 ± 0.04
*p‐*Value (vs. baseline)^a^			
Test product	30		*<0.001*
Non‐treatment control	30		*0.199*
*p‐*Value (vs. control)^b^			
Test product			*<0.001*

*Note*: *N* means the data size for data calculation.

Abbreviation: SE, standard error.

^a^ Between time‐points, use paired samples test with 0.05 significance level, *p*–value < 0.05, the results observed very significant.

^b^ Between treatments, use an independent samples test with 0.05 significance level, *p*–value < 0.05, the results observed very significant.

**FIGURE 1:** Gloss—between time‐point.

**FIGURE 2:** Gloss—between treatment.

An increased value indicates greater glossiness, and it was observed that glossiness improved signficantly from 2.90 ± 0.02 at T0 to 3.38 ± 0.02 at T1, following a single application of the test product. The percentage of mean change from the baseline of glossiness of hair bundles was 16.42%.

Compared with the non‐treatment control, the test product revealed significantly better efficacy in improving glossiness of hair bundles after a single application.

The sensory evaluator assessed the difference in glossiness between the test group baseline and non‐treatment control group (T0–NT) and that after‐test product application (T1–NT). The larger the difference between after‐test product application and baseline, the better the gloss improvement. The experimental results are displayed in Table 2 and Figures 3 and 4.

**TABLE 2:** Gloss—sensory assessment.

		Time‐point	
	*N*	T0–NT (baseline)	T1–NT
Mean ± SE	30	0.13 ± 0.08	0.60 ± 0.10
Change from baseline (mean ± SE)	30		0.47 ± 0.13
Percentage of improvement^a^	30		63.33%
*p‐*Value (vs. baseline) ^b^	30		*0.002*

*Note*: *N* means the data size for data calculation.

Abbreviations: NT, non‐treatment; SE, standard error.

^a^ Percentage of improvement = [count that (T1–TN) – (T0–TN) is greater than 0]/30 × 100%.

^b^ Between time‐points, use Wilcoxon signed ranks test with 0.05 significance level, *p*–value < 0.05, the results observed very significant.

**FIGURE 3:** Gloss‐sensory assessment between time‐point.

**FIGURE 4:** Improvement ratio of gloss‐sensory assessment.

According to the gloss sensory evaluation results, we found that the difference between the test group and the non‐treatment control group was significantly improved between T0 and T1 after the test product single application. It was improved from 0.13 ± 0.08 at T0 to 0.60 ± 0.10 at T1.

The article "Comparative study of instrumental measurement and sensory evaluation methods for the repairing effect of mildly damaged hair bundles" was published in 2023. Journal: Skin Res Technol.

At the same time, 63.33% of the samples in the test group demonstrated improvement compared to the corresponding non‐treatment control group, which was larger than the proportion of non‐improvement. This indicates that the hair bundle gloss improvement rate in the test group was higher than that in the non‐treatment control group.

### 3.2 Results of friction performance

Instrumental measurement results showed that the larger the difference after the test product application (T1) and baseline (T0), the better the improvement in friction performance (friction coefficient and friction work). The results are presented in Tables 3 and 4 and Figures 5, 6, 7, 8.

**TABLE 3:** Friction coefficient—instrumental measurement.

		Along hair cuticle		Against hair cuticle	
	*N*	T0 (baseline)	T1	T0 (baseline)	T1
Mean ± SE					
Test product	30	0.44 ± 0.02	0.24 ± 0.01	1.04 ± 0.03	0.57 ± 0.02
Non‐treatment control	30	0.45 ± 0.02	0.40 ± 0.01	1.08 ± 0.02	1.01 ± 0.03
Change from baseline (mean ± SE)					
Test product	30		–0.21 ± 0.02		–0.47 ± 0.04
Non‐treatment control	30		–0.05 ± 0.02		–0.07 ± 0.03
*p‐*Value (vs. baseline)^a^					
Test product	30		*<0.001*		*<0.001*
Non‐treatment control	30		*0.015*		*0.052*
*p‐*Value (vs. control)^b^					
Test product			*<0.001*		*<0.001*

*Note*: *N* means the data size for data calculation.

Abbreviation: SE, standard error.

^a^ Between time‐points, use paired samples test with 0.05 significance level, *p*–value < 0.05, the results observed very significant.

^b^ Between treatments, use an independent samples test with 0.05 significance level, *p*–value < 0.05, the results observed very significant.

**TABLE 4:** Friction work—instrumental measurement.

		*N*	Along hair cuticle		Against hair cuticle	
			T0 (baseline)	T1	T0 (baseline)	T1
Mean ± SE	Test product	30	0.03 ± 0.00	0.01 ± 0.00	0.06 ± 0.00	0.03 ± 0.00
	Non‐treatment control	30	0.03 ± 0.00	0.02 ± 0.00	0.06 ± 0.00	0.06 ± 0.00
Change from baseline (mean ± SE)	Test product	30		–0.01 ± 0.00		–0.03 ± 0.00
	Non‐treatment control	30		0.00 ± 0.00		0.00 ± 0.00
*p‐*Value (vs. baseline)^a^	Test product	30		*<0.001*		*<0.001*
	Non‐treatment control	30		*0.013*		*0.045*
*p‐*Value (vs. control)^b^	Test product			*<0.001*		*<0.001*

*Note*: *N* means the data size for data calculation.

Abbreviation: SE, standard error.

^a^ Between time‐points, use paired samples test with 0.05 significance level, *p*–value < 0.05, the results observed very significant.

^b^ Between treatments, use an independent samples test with 0.05 significance level, *p*–value < 0.05, the results observed very significant.

The article "Comparative study of instrumental measurement and sensory evaluation methods for the repairing effect of mildly damaged hair bundles" was published in 2023. Journal: Skin Res Technol.

**FIGURE 5:** Friction coefficient—between time‐point.

**FIGURE 6:** Friction coefficient—between treatment.

**FIGURE 7:** Friction work—between time‐point.

**FIGURE 8:** Friction work—between treatment.

By analyzing the data of friction coefficient, a lower value indicates smoother hair bundles, and the friction coefficient of the hair cuticle improved from 0.44 ± 0.02 at T0 to 0.24 ± 0.01 at T1; there was a significant improvement between T0 and T1 after the test product was applied. The percentage of mean change from baseline of the friction coefficient along the hair cuticle was 46.61%. The friction coefficient against hair cuticle was improved from 1.04 ± 0.03 at T0 to 0.57 ± 0.02 at T1; there was a significant improvement between T0 and T1 after the test product single application and the percentage of mean change from baseline of friction coefficient against the hair cuticle was 45.59%.

Compared to the non‐treatment control, the test product demonstrated significantly better efficacy in improving along and against the hair cuticle friction coefficient after a single application.

By analyzing the data of friction work, a lower value means smoother hair bundles, the friction work along hair cuticle was improved from 0.03 ± 0.00 at T0 to 0.01 ± 0.00 at T1, and there was a significant improvement between T0 and T1 after the test product single application. The percentage of mean change from baseline of friction work along the hair cuticle was 46.53%. The friction work against hair cuticle was improved from 0.06 ± 0.00 at T0 to 0.03 ± 0.00 at T1; there was an improvement with significance between T0 and T1 after the test product single application and the percentage of mean change from the baseline of friction work against hair cuticle was 45.31%.

Compared to the non‐treatment control, the test product displayed significantly better efficacy in improving the along and against hair cuticle friction work in a single application.

The sensory evaluator assessed the difference in smoothness between the test group baseline and non‐treatment control group (T0–NT) and after‐test product application (T1–NT). The larger the difference between the test product application and the baseline, the better the smoothness improvement. The experimental results are displayed in Table 5 and Figures 9 and 10.

**TABLE 5:** Smoothness—sensory assessment.

		Time‐point	
	*N*	T0–NT (baseline)	T1–NT
Mean ± SE	30	–0.05 ± 0.14	0.52 ± 0.16
Change from baseline (mean ± SE)	30		0.57 ± 0.19
Percentage of improvement^a^	30		60.00%
*p‐*Value (vs. baseline)^b^	30		*0.012*

*Note*: *N* means the data size for data calculation.

Abbreviations: NT, non‐treatment; SE, standard error.

^a^ Percentage of improvement = [count that (T1–TN) – (T0–TN) is greater than 0]/30 × 100%.

^b^ Between time‐points, use Wilcoxon signed ranks test with 0.05 significance level, *p*–value < 0.05, the results observed very significant.

The article "Comparative study of instrumental measurement and sensory evaluation methods for the repairing effect of mildly damaged hair bundles" was published in 2023. Journal: Skin Res Technol.

**FIGURE 9:** Smoothness‐sensory assessment between time‐point.

**FIGURE 10:** Improvement ratio of smoothness‐sensory assessment.

According to the smoothness‐sensory evaluation results, the difference between the test group and the non‐treatment control group was significantly improved between T0 and T1 after the test product single application. It was improved from −0.05 ± 0.14 at T0 to 0.52 ± 0.16 at T1. Sixty percent of the samples demonstrated an improvement in the sensory evaluation difference between the test group and the non‐treatment control group, which was larger than the proportion of non‐improvement, indicating that the rate of improvement in the smoothness of the test group was higher than that of the non‐treatment control group.

### 3.3 Correlation between instrumental measurement and sensory assessment

The correlation coefficient between instrument measurement and sensory assessment was 0.838 for gloss parameter, 0.895 for friction OUT (with the grain of hair) coefficient, 0.895 for friction OUT WORK DONE, 0.850 for friction RTN (against the grain of hair) coefficient, and 0.851 for friction RTN WORK DONE. The correlation coefficients between instrument measurements and sensory assessments were all greater than 0.800. The experimental results are displayed are displayed in Tables 6 and 7 and Figures 11 and 12.

**TABLE 6:** Correlation coefficient of glossiness.

Gloss parameter			Instrument measurement (T1–T0)
Spearman's rho	Sensory assessment (T1–T0)	Correlation coefficient	0.838^a^
		Significance (two‐tailed)	0.000
		*N*	30

^a^ Correlation is significant at the 0.01 level (two‐tailed).

**TABLE 7:** Correlation coefficient of friction (COF) performance.

Smoothness parameter			COF OUT (T1–T0)	WORK DONE OUT (T1–T0)	COF RTN (T1–T0)	WORK DONE RTN (T1–T0)
Spearman's rho	Sensory assessment (T1–T0)	Correlation coefficient	0.895^a^	0.895^a^	0.850^a^	0.851^a^
		Significance (two‐tailed)	*0.000*	*0.000*	*0.000*	*0.000*
		*N*	30	30	30	30

^a^ Correlation is significant at the 0.01 level (two‐tailed).

**FIGURE 11:** Correlation of gloss parameters.

**FIGURE 12:** Correlation of friction parameters.

## 4 DISCUSSION

The gloss and friction properties of hair bundles are the most intuitive parameters to depict the condition of the hair cuticle, considering that the improvement of the hair cuticle state is the focus of repair efficiency. The results of this research depict that both the instrument test and sensory evaluation are consistent, suggesting that instrumental testing can effectively verify the repair function of hair bundle care products and provide objective evidence for the hair care product repair function test bundle. Therefore, instrument measurements are also applicable and scientific for evaluating the friction performance of hair bundles. In addition, the instrument test is convenient to operate, less time‐consuming, unlimited by the fatigue of evaluators or recruitment of subjects, and can be operated at large hair cuticles, which can greatly improve the screening and adjustment speed in the early stages of hair care product formulation development.

The article "Comparative study of instrumental measurement and sensory evaluation methods for the repairing effect of mildly damaged hair bundles" was published in 2023. Journal: Skin Res Technol.

At the present stage, only a single product and non‐treatment control were tested to verify whether the product had a therapeutic effect. Further studies are needed to determine whether this test method can be used for cross‐sectional comparisons of product efficacy, to analyze the differences between products and whether the type, formulation, or other factors affect the accuracy of the instrument test results.

In order to make the display of product effects more suitable for consumers to understand while ensuring the scientificity of its data results, this article combines quantitative means of subjective observation and objective measurement to further provide an application model that can be quickly and accurately applied. In addition, scientifically extracting the supporting basis for the efficacy claim required by the product reduces the possible errors in subjective observation and at the same time improves the shortcomings of the original microscopic science and technology that cannot be quickly replicated due to its precision.

   

## Data Availability

Data sharing is not applicable to this article as no datasets were generated or analyzed during the current study.
